The article "Design of Automated Deep Learning-Based Fusion Model for Copy-Move Image Forgery Detection" was retracted in 2023. Reasons: signs of a paper mill; suspected computer-generated content; unreliable results or conclusions; concerns about the data.

# Design of Automated Deep Learning-Based Fusion Model for Copy-Move Image Forgery Detection

**DOI:** 10.1155/2022/8501738

**Published:** 2022-01-31

**Authors:** N. Krishnaraj, B. Sivakumar, Ramya Kuppusamy, Yuvaraja Teekaraman, Amruth Ramesh Thelkar

**Affiliations:** ^1^Department of Networking and Communications, School of Computing, SRM Institute of Science and Technology, Kattankulathur 603203, Chennai, India; ^2^Department of Computing Technologies, School of Computing, SRM Institute of Science and Technology, Kattankulathur 603203, Chennai, India; ^3^Department of Electrical and Electronics Engineering, Sri Sairam College of Engineering, Bangalore 562106, Karnataka, India; ^4^Department of Electronic and Electrical Engineering, The University of Sheffield, Sheffield S1 3JD, UK; ^5^Faculty of Electrical & Computer Engineering, Jimma Institute of Technology, Jimma University, Jimma, Ethiopia

## Abstract

Due to the exponential growth of high-quality fake photos on social media and the Internet, it is critical to develop robust forgery detection tools. Traditional picture- and video-editing techniques include copying areas of the image, referred to as the copy-move approach. The standard image processing methods physically search for patterns relevant to the duplicated material, restricting the usage in enormous data categorization. On the contrary, while deep learning (DL) models have exhibited improved performance, they have significant generalization concerns because of their high reliance on training datasets and the requirement for good hyperparameter selection. With this in mind, this article provides an automated deep learning-based fusion model for detecting and localizing copy-move forgeries (DLFM-CMDFC). The proposed DLFM-CMDFC technique combines models of generative adversarial networks (GANs) and densely connected networks (DenseNets). The two outputs are combined in the DLFM-CMDFC technique to create a layer for encoding the input vectors with the initial layer of an extreme learning machine (ELM) classifier. Additionally, the ELM model's weight and bias values are optimally adjusted using the artificial fish swarm algorithm (AFSA). The networks' outputs are supplied into the merger unit as input. Finally, a faked image is used to identify the difference between the input and target areas. Two benchmark datasets are used to validate the proposed model's performance. The experimental results established the proposed model's superiority over recently developed approaches.

## 1. Introduction

Recently, the extension of Internet services and the strengthening and proliferation of social networks such as Reddit, Facebook, and Instagram had had an important effect on the number of content prevailing in digital media. As per the International Telecommunication Union (ITU), by the end of 2019, 53.6% of the world's population utilizes the Internet, which implies around 4.1 billion peoples have access to these technologies, as well as with distinct mechanisms accessed on the Internet [1]. Even though in many situations has only been manipulated or content shared is original for entertainment purposes only, in another case the manipulation might be intended for falsehood purposes, using forensic and political consequences, for example, utilizing the false contents as digital proof in criminal investigations. Video/Image manipulation represents few actions that are accomplished on the digital content via software editing tools (e.g., GIMP, PIXLR, Adobe Photoshop) or artificial intelligence. Especially, the copy-move techniques copy a portion of the image and paste it onto similar images [2]. Since editing tools advance, the quality of false images rises and it seems to be original images. Furthermore, postprocessing manipulations, such as brightness equalization/changes and JPEG compression, might decrease the traces left by manipulation and make it very complex to identify [3]. The copy-move forgery detection (CMFD) consists of deep learning- and hand-crafted-based approaches. The previous one is largely separated into hybrid, block, and key point-based methods and next employs convention framework from fine-tuned/scratch algorithms.

The article "Design of Automated Deep Learning-Based Fusion Model for Copy-Move Image Forgery Detection" was retracted in 2023. Reasons: signs of a paper mill; suspected computer-generated content; unreliable results or conclusions; concerns about the data.

Block-based methods utilized distinct kinds of feature extraction, for example, Tetrolet transforms/Fourier transform, and DCT (discrete cosine transform). The major concern is the performance reduction while the copied objects are resized/rotated since the recognition of forging can be performed by a matching procedure [4]. Conversely, key point-based methods such as SURF (Speed-Up Robust Features) and SIFT (scale-invariant feature transform) are very stronger to lighting and rotation differences; however, they have many problems to conquer, for example, natural duplicate objects spotted as false duplicate objects and reliance on original key point in an image, and detect forgeries in the area of uniform intensity [5]. A hybrid method provides constant results by means of F1-score, precision (P), and recall (R) for an individual dataset.

### 1.1. Motivation

There is a current development of deviating traditionally handcrafted feature extraction for employing convolutional neural network (CNN)-based extractor. But, in few conventional CNN-based forensic detectors is usually not real world for several details, for example, by means of strength in feature extraction and solution of tampering position. Thus, there are various attempts to develop a preprocessing layer for enhancing the strength of feature extraction [6] and combine several detector-based likelihood maps and individual CNN-based consistency maps for improving the solution of tampering location. But still, they endure numerous limits in the abovementioned methods. Initially, current pixel-wise tampering detector adapts an autonomous patch-based approach instead of utilizing the related data amongst patches [7]. Moreover, the lack of statistical features on flat regions (blue ocean, clear sky, and so on) leads to uncertainty approximation and degradation of recognition accuracy. In this situation, the texture of an image content has become a decisive factor to enhance recognition performance. In addition, with the quick growth of image-editing software, the remainder left by the manipulation process has behavior like its pristine versions (viz., tampering trace is difficult to identify) [8]. Then, decreasing the possibility of recognition mismatch and enhancing the solution of localization (managed by the small units of finding) still remain an open challenge.

The article "Design of Automated Deep Learning-Based Fusion Model for Copy-Move Image Forgery Detection" was retracted in 2023. Reasons: signs of a paper mill; suspected computer-generated content; unreliable results or conclusions; concerns about the data.

### 1.2. Scope of the Research Work

This article presents an automated DL-based fusion model for copy-move forgery detection and localization (DLFM-CMDFC). The proposed DLFM-CMDFC technique comprises the fusion of generative adversarial network (GAN) and densely connected network (DenseNet) models.

## 2. Related Works

Yao et al. [9] develop efficient detectors, which can complete image fake localization and detection. Particularly, based on the developed continuous high-pass filter, they initially determine an effective CNN framework automatically for and adaptively extracting features and propose an RFM model for improving tamper recognition performance and localization solution. Abdalla et al. [10] examine copy-move counterfeit findings with a fusion processing method including an adversarial method and deep convolution method. Four databases were employed. The result indicates a considerably higher recognition accuracy (∼95%) shown by the discriminator counterfeit detector and DL-CNN models. Accordingly, an end-to-end trained DNN method for counterfeit finding seems to be an optimum approach.

Diallo et al. [11] introduce an architecture enhancing strength for image counterfeit recognition. The vital stage of this architecture is to consider the image quality matching to the selected application. Consequently, it is based on a camera recognition method-based CNN model. Lossy compressions like JPEG are taken into account as general kind of inadvertent/intentional concealment of image counterfeit, which results in manipulation. Consequently, the trainable CNN is fed into a combination of distinct amounts of uncompressed and compressed images. Rodriguez-Ortega et al. [12] present 2 methods, which utilize the DL method, an approach with a convention framework, and a method with the TL model. In all the cases, the effect of depth of the network can be examined by means of F1-score, precision (P), and recall (R). In addition, the challenge of generalization can be resolved from 8 distinct open-access databases.

The article "Design of Automated Deep Learning-Based Fusion Model for Copy-Move Image Forgery Detection" was retracted in 2023. Reasons: signs of a paper mill; suspected computer-generated content; unreliable results or conclusions; concerns about the data.

In the study by Doegar et al. [13], CNN-based pretrained AlexNet method deep feature was employed, which is effective and efficient than that of current advanced methods on open-source standard database MICC-F220. Marra et al. [14] introduce a CNN-based image counterfeit recognition architecture that makes decisions according to the full resolution data collected from the entire image. Because of gradient checkpointing, the architecture can be trained end to end using constrained memory resources and weak (image-level) supervision, which enables the joint optimization of each parameter.

Dixit and Bag [15] presented a technique where SWT and spatial-limited edge-preserving watershed segmentation are employed on input images in the preprocessing phase. Descriptor computation and key point extraction were implemented. Outlier removal can be executed by the RANSAC approach. Furthermore, counterfeit areas are positioned by relation map generation. In Bi et al. [16], a counterfeit localization generator GM has been presented on the basis of a multidecoder single task method. Through adversarial training 2 generators, the presented alpha-learnable WCT blocks in GT suppress manually the tampering artifact in the counterfeit images. In the meantime, the localization and detection capacities of GM would be enhanced by learning the phony images restored by GT.

Ghai et al. [17] aim at designing a DL-based image counterfeit recognition architecture. The presented model focuses on detecting images counterfeit with splicing and copy-move methods. The image conversion method supports the detection of related features to the network for training efficiently. Next, the pretrained personalized CNN is utilized for training the public standard databases. In Rao et al. [18], a new image counterfeit localization and detection system has been presented on the basis of the DCNN model that integrates a multisemantic CRF-based attention method. The presented model depends on the main findings that the boundary transition artifact arising from the blending operation is global in several image counterfeit manipulations, that is, established in this model using a method with CRF-based attention method through making attention mapping to characterize the possibility of being counterfeit for all the pixels in an image.

The article "Design of Automated Deep Learning-Based Fusion Model for Copy-Move Image Forgery Detection" was retracted in 2023. Reasons: signs of a paper mill; suspected computer-generated content; unreliable results or conclusions; concerns about the data.

## 3. The Proposed Model

In this study, an efficient DLFM-CMDFC technique is presented for automated copy-move forgery detection and localization model. The proposed DLFM-CMDFC technique encompasses the fusion of GAN and DenseNet models. In DLFM-CMDFC technique, the two outcomes are combined into a layer to define the input vectors with the initial layer of the ELM classifier. Moreover, the optimal parameter tuning of the ELM model takes place by the use of AFSA. The outcomes of the networks are fed as input to the merger unit. Lastly, the difference between the input and targets areas is identified in a forged image.

### 3.1. GAN-Based Forgery Image Generation

Advancements of technology are assisting GAN to generate forged images, which fool even the more advanced detector [58]. It must be noted that the main objective of generative adversarial network is to create images that could not be differentiated from the primary source image. As demonstrated, generator *G*_*A*_ was applied for transforming input images A from domain *D*_*A*_ to output domain *D*_*B*_. Then, generator *G*_*B*_ can be utilized for mapping image *B* back to domain *D*_*A*_ (the original domain). Thereby, another set of cycle consistency losses are included in the standard adversarial losses borne by the discriminator, therefore, attaining *A*=*G*(*G*(*A*)) and assisting the 2 images to be coupled. Highly advanced editing tools are needed for changing an image context. This tool should be capable of altering images when preserving the original source perspectives, shadowing, etc. Those without forgery detection training will not able to differentiate the actual image from an image forged utilizing this methodology that implies that it is the best candidate to develop support material for false news reports.

GAN task is given in the following: (1) build a discriminator network; (2) load a dataset; (3) generate a sample image; (4) build a generator network; (5) closing thoughts; (7) training difficulties. The GAN network branch is shown in Figure 1 [19].

In the presented GAN network, it is considered 2 major phases: (1) in the initial phase, the generator fashions an image from haphazard noise input, and (2) then, the image, as well as various images based on a similar database, is proposed for the discriminator. (3) After the discriminator is proposed by the real and forged images, it provides likelihoods through numbers in the range of zero and one, extensive. Now, zero denotes a forged image and one represents a higher probability for validity. It should be noted that the discriminator must be pretrained previous to the generator since it generates clear gradients. Retaining the constant values enables the network to possess a good understanding of the gradients, that is, the foundation of its learning. But GAN has been proposed as a kind of game performed among opposite networks, and retaining their balance could be problematic. Inopportunely, learning is hard for GAN when the generator/discriminator is highly proficient since GAN usually needs extensive training time. Thus, for example, a GAN can take a long time for an individual GPU, whereas for an individual CPU, a GAN might need few more days.

The article "Design of Automated Deep Learning-Based Fusion Model for Copy-Move Image Forgery Detection" was retracted in 2023. Reasons: signs of a paper mill; suspected computer-generated content; unreliable results or conclusions; concerns about the data.

### 3.2. DenseNet Model

In this study, the DenseNet-121 framework is utilized as the foundation. In addition, the transfer learning method has been employed in the DenseNet architecture for enhancing the system performance [20]. DenseNets in contrast to common belief require fewer parameters when compared to traditional CNN models since they do not want to learn unnecessary feature maps. The basic idea of the DenseNet architecture is the feature reuse that leads to tremendously compact version. Consequently, it requires fewer parameters when compared to another CNN model because no feature map is repeated. Once CNN goes further, it faces challenges. DenseNet makes this connectivity much easier by simply interconnecting all the layers straightforwardly with every layer. DenseNets utilize the network's capability by reutilizing features. All the layers in DenseNet obtain further input over every prior layer and transmit its feature map to the succeeding layers.

All the layers receive good understanding from the above layers, namely, the idea of concatenation that is utilized. For maximizing computational recycling among the classifiers, incorporating several classifiers to a model and DCNN and interconnect with dense connectivity for effective image classification [21]. A study has proved that a convolution network with smaller connections among layers and those nearer to the output could be very much deeper, and it would be more precise for training. DenseNet attains important developments over the advanced technology when consuming minimum memory and processing to improve its efficiency. The DL library PyTorch and torchvision are utilized, that is, a pretrained data learning method that contains a maximal control across overfitting and also improves the optimization of results from the very first. It consists of 1 classification layer (16), 2 DenseBlocks (1 × 1 and 3 × 3 convs), 3 transition layers (6, 12, and 24), and 5 convolution and pooling layers.

### 3.3. Optimal ELM Model Using AFSA

ELM is essentially an SLFN algorithm. The variance among ELM and SLFN exists within the weight of the output layer, and hidden layer neurons are upgraded. In SLFN, the weight of input and output layers is initiated arbitrarily, and the weight of the layers is upgraded using the BP model. In ELM, the weight of the hidden layer is allocated arbitrarily but not upgraded, and the weight of the output layer is upgraded at the time of training. Since in ELM, the weight of single layer is upgraded against both layers of SLFN, it would make ELM quicker when compared to SLFN.

The article "Design of Automated Deep Learning-Based Fusion Model for Copy-Move Image Forgery Detection" was retracted in 2023. Reasons: signs of a paper mill; suspected computer-generated content; unreliable results or conclusions; concerns about the data.

Assume the trained database as (*x*_*j*_, *t*_*j*_) in which *x*_*j*_=[*x*_*j*1_, *x*_*j*2_,   …,*x*_*jN*_]^*T*^ represents the input vector and *t*_*j*_ denotes the output vector. The output of *j*^th^ hidden layer neuron is represented as *g*(*w*_*i*_, *b*_*i*_, *x*_*j*_), in which *w*_*i*_ indicates the weight vector connected the input neuron to *i*^th^ hidden layer neuron, *b*_*i*_ signifiers the bias of *i*^th^ hidden neurons, and *g* denotes the activation function. All the hidden layer neurons of ELM are interconnected to all the output layer neurons with related weight, and they represent the weight interconnecting the *i*^th^ hidden layer neuron with output neuron as *β*_*i*_. This framework is denoted arithmetically by

(1) $$\begin{array}{c} \sum_{i=1}^{L}\beta_{i}g\left(w_{i},b_{i},x_{j}\right)=t_{j}, \end{array}$$

where *L* represents the number of hidden neurons, and *j* indicates the output or input sample of overall *N* trained samples. The aforementioned formula is expressed by

(2) $$\begin{array}{c} H\beta =T. \end{array}$$

In the above formula, consider *m* output node as

(3) $$\begin{array}{c} \beta ={\left[\begin{array}{c} \beta_{1}^{T}\\ \vdots \\ \beta_{L}^{T} \end{array}\right]}_{L\times m}\;\mathrm{and}\;T={\left[\begin{array}{c} t_{1}^{T}\\ \vdots \\ t_{N}^{T} \end{array}\right]}_{N\times m}, \end{array}$$

where *H* denotes the output matrix of the hidden layer, which is given as

(4) $$\begin{array}{c} H=\left[\begin{array}{ccc} g\left(w_{1},b_{1},x_{1}\right) & \cdots & g\left(w_{\text{L}},b_{\text{L}},x_{1}\right)\\ \vdots & \ddots & \vdots \\ g\left(w_{1},b_{1},x_{N}\right) & \cdots & g\left(w_{\text{L}},b_{\text{L}},x_{N}\right) \end{array}\right]. \end{array}$$

The minimum norm least square of (2) is

(5) $$\begin{array}{c} \hat{\beta }=H^{+}T, \end{array}$$

where *H*^+^ is the Moore–Penrose generalized inverse of matrix *H*. *H*^+^ is evaluated by singular value decomposition (SVD), QR approach, orthogonal projection model [22], and orthogonalization method.

It must standardize the scheme (to avoid overfitting), and the optimization issues turn into

(6) $$\begin{array}{c} \text{min}\left({\left\|\beta \right\|}^{2}+C\sum_{i=1}^{N}{\left\|\xi_{i}^{T}\right\|}^{2}\right), \end{array}$$

where *ξ*_*i*_=*t*_*i*_^*T*^ − *h*(*x*_*i*_)*β* denotes the trained error of *i*^th^ instance and *C* denotes the appropriate penalty factor. It might convert these problems to its dual form and create the Lagrangian function as

(7) $$\begin{array}{c} F={\left\|\beta \right\|}^{2}+C\sum_{i=1}^{N}{\left\|\xi \right\|}^{2}-\sum_{i=1}^{N}\sum_{j=1}^{L}\alpha_{ij}\left(h\left(x_{i}\right)\beta_{j}-t_{ij}+\xi_{ij}\right). \end{array}$$

Take the partial derivative of the aforementioned formula and apply KKT condition. When *L* < *N*, the size of matrix *H*^*T*^*H* is lesser when compared to matrix *HH*^*T*^,

(8) $$\begin{array}{c} \beta =H^{+}T={\left(\frac{I}{C}+H^{T}H\right)}^{-1}H^{T}T. \end{array}$$

Hence, the last output of ELM is

(9) $$\begin{array}{c} f\left(x\right)=h\left(x\right)\beta =h\left(x\right){\left(\frac{I}{C}+H^{T}H\right)}^{-1}H^{T}T. \end{array}$$

Once *L*≻*N*, the size of matrix *HH*^*T*^ is lesser when compared to the matrix *H*^*T*^*H*, the solution of the equation becomes

(10) $$\begin{array}{c} \beta =H^{+}T=H^{T}{\left(\frac{I}{C}+HH^{T}\right)}^{-1}T. \end{array}$$

Thus, the last output of ELM is

(11) $$\begin{array}{c} f\left(x\right)=h\left(x\right)\beta =h\left(x\right)H^{T}{\left(\frac{I}{C}+HH^{T}\right)}^{-1}T. \end{array}$$

For the binary classification problems, the decision function of ELM can be expressed by

(12) $$\begin{array}{c} f\left(x\right)=\text{sign}\left(h\left(x\right)\beta \right). \end{array}$$

For multiclass instance, the class label of instance is expressed by

(13) $$\begin{array}{c} \text{label}\left(x\right)=\underset{1\leq i\leq m}{\text{arg max}}\left\{f_{i}\left(x\right)\right\}. \end{array}$$

Then

(14) $$\begin{array}{c} f\left(x\right)={\left.r_{1}\left(x\right),f_{2}\left(x\right),f_{3}\left(x\right),\ldots ,f_{n}\left(x\right)\right]}^{T}. \end{array}$$

ELM was employed for the classification and prediction tasks in various fields. To optimally adjust the learning rate of the ELM model, the AFSA is used, which is a kind of swarm intelligence method depending on the behavior of the animal. It was developed by Li et al. in 2002 [23]. Its fundamental is the inspiration of collision, foraging, and clustering behavior of fish and the collective support in a fish swarm for realizing a global optimum points. The highest distance pass through in the artificial fish method can be determined by *Step*, the apparent distance pass through by the artificial fish can be determined by *Visual*, the retry amount represent the Try_−_*Number* also the factors of crowd amount represent *η*. The location of a single artificial fish is defined by the resulting vectors *X*=(*X*_1_, *X*_2_,…, *X*_*n*_), and the distance among artificial fish *i* and *j* denotes *d*_*ij*_=|*X*_*i*_ − *X*_*j*_|. The behavior function for the artificial fish can be determined by random, prey, swarm, and follow.

The article "Design of Automated Deep Learning-Based Fusion Model for Copy-Move Image Forgery Detection" was retracted in 2023. Reasons: signs of a paper mill; suspected computer-generated content; unreliable results or conclusions; concerns about the data.

Assume that the fish observe their food using their eyes and the present location is *X*_*i*_, as well as an arbitrarily elected location is *X*_*j*_ within their perceptive range:

(15) $$\begin{array}{c} X_{j}=X_{i}+\text{Visual }\times \text{rand}\left(0∼1\right), \end{array}$$

where *rand* (0‐1) represents an arbitrary value between zero and one. When *Y*_*i*_ > *Y*_*j*_, the fish move in this direction. Or else, the method arbitrarily selects a novel location *X*_*j*_ for judging whether it fulfills the moving criteria. When it performs,

(16) $$\begin{array}{c} X_{i}^{t+1}=X_{i}^{t}+\frac{X_{j}-X_{i}^{t}}{\left\|X_{j}-X_{i}^{t}\right\|}\times \text{Step}\times \text{rand}\left(0∼1\right). \end{array}$$

When it does not Try_−_*Number* times, an arbitrary movement can be generated by

(17) $$\begin{array}{c} X_{i}^{t+1}=X_{i}^{t}+\text{Visual}\times \text{rand}\left(0∼1\right). \end{array}$$

In order to prevent overcrowding, an artificial present location *X*_*i*_ is fixed. Next, the amount of fish in its *n*_*f*_ company and *X*_*c*_ center in the region (i.e., *d*_*ij*_ < *Visual*) are defined. When *Y*_*c*_/*n*_*f*_ < *η* × *Y*_*i*_, the position of companion represents the optimal number of food and lower crowding. Subsequently, the fish moves to its companion region center position:

(18) $$\begin{array}{c} X_{i}^{t+1}=X_{i}^{t}+\frac{X_{c}-X_{i}^{t}}{\left\|X_{c}-X_{i}^{t}\right\|}\times \text{Step}\times \text{rand}\left(0∼1\right). \end{array}$$

Or else it starts to perform the behavior of prey.

The present location of artificial fish swarm can be determined by *X*_*i*_. The swarm defines its main company *Y*_*j*_ as *X*_*j*_ in the region (i.e., *d*_*ij*_ < Visual). When *Y*_*j*_/*n*_*f*_ < *η* × *Y*_*i*_, the position of companies represents the optimal number of food and lesser crowd [24]. Next, the swarm moves to *X*_*j*_:

(19) $$\begin{array}{c} X_{i}^{t+1}=X_{i}^{t}+\frac{X_{j}-X_{i}^{t}}{\left\|X_{j}-X_{i}^{t}\right\|}\times \text{Step}\times \text{rand}\left(0∼1\right). \end{array}$$

It enables artificial fish to attain company and food through a large regional area. A location is arbitrarily chosen, as well as artificial fish moves to it.  Figure 2 illustrates the flowchart of AFSA.

With the searching space of *D*  dimensional, highly probable distance amid 2 artificial fishes is utilized for vigorously limiting the *Visual* & *Step* of an artificial fish. It is determined by Max*D*:

(20) $$\begin{array}{c} \text{Max}D\;=\sqrt{{\left(x_{\text{max}}-x_{\text{min}}\right)}^{2}\times D}, \end{array}$$

where  *x*_min_ and *x*_max_ represent the lower and upper bounds of the optimization range, respectively, and *D* indicates the dimension of the search space.

The article "Design of Automated Deep Learning-Based Fusion Model for Copy-Move Image Forgery Detection" was retracted in 2023. Reasons: signs of a paper mill; suspected computer-generated content; unreliable results or conclusions; concerns about the data.

## 4. Experimental Validation

This section investigates the result analysis of the proposed model on MNIST and COCO datasets.  Figure 3 shows a few sample image, tampered image, and localization image.

Table 1 and Figure 4 provide the performance analysis of the proposed model on the applied MNIST dataset under varying runs. The results demonstrated that the proposed model has gained effective outcomes under distinct runs. For instance, under run-1, the proposed model has attained effective outcome with the prec_*n*_ of 96.38%, rec_*l*_  of 93.71%, acc_*y*_ of 94.29%, and *F*_score_ of 95.98%. Also, under run-3, the presented manner has reached effective outcome with the prec_*n*_ of 93.54%, rec_*l*_  of 97.30%, acc_*y*_ of 94.88%, and *F*_score_ of 97.19%. Besides, under run-5, the presented technique has obtained effective outcome with the prec_*n*_ of 96.80%, acc_*y*_ of 97.43%, acc_*y*_ of 96.87%, and *F*_score_ of 94.69%.

Figure 5 demonstrates the ROC analysis of the DLFM-CMDFC technique on the test MNIST dataset. The figure has shown that the DLFM-CMDFC technique has resulted in an effective outcome with a maximum ROC of 98.5180.

Figure 6 portrays the accuracy analysis of the DLFM-CMDFC technique on the test MNIST dataset. The results demonstrated that the DLFM-CMDFC technique has accomplished improved performance with increased training and validation accuracy. It is noticed that the DLFM-CMDFC technique has gained improved validation accuracy over the training accuracy. Similarly, Figure 7 depicts the loss analysis of the DLFM-CMDFC technique on the test MNIST dataset. The results established that the DLFM-CMDFC technique has resulted in a proficient outcome with reduced training and validation loss. It is observed that the DLFM-CMDFC technique has offered reduced validation loss over the training loss.

Table 2 and Figure 8 offer the performance analysis of the presented technique on the applied CIFAR-10 dataset under varying runs. The outcomes exhibited that the presented approach has reached effectual outcomes under different runs. For instance, under run-1, the presented manner has attained effective outcome with the prec_*n*_ of 96.52%, rec_*l*_  of 96.15%, acc_*y*_ of 96.36%, and *F*_score_ of 96.66%. Followed by, under run-3, the proposed model has attained effective outcome with the prec_*n*_ of 97.95%, rec_*l*_  of 96.68%, acc_*y*_ of 97%, and *F*_score_ of 96.57%. In addition, under run-5, the projected system has achieved effective outcome with the prec_*n*_ of 97.46%, rec_*l*_  of 96.50%, acc_*y*_ of 97.35%, and *F*_score_ of 94.52%.

The article "Design of Automated Deep Learning-Based Fusion Model for Copy-Move Image Forgery Detection" was retracted in 2023. Reasons: signs of a paper mill; suspected computer-generated content; unreliable results or conclusions; concerns about the data.

Figure 9 depicts the ROC analysis of the DLFM-CMDFC technique on the test CIFAR-10 dataset. The figure outperformed that the DLFM-CMDFC scheme has resulted in an effective outcome with the maximal ROC of 98.7262.

Figure 10 demonstrates the accuracy analysis of the DLFM-CMDFC technique on the test CIFAR-10 dataset. The outcomes showcased that the DLFM-CMDFC technique has accomplished improved efficiency with increased training and validation accuracy. It can be noticed that the DLFM-CMDFC manner has gained increased validation accuracy over the training accuracy.

Figure 11 represents the loss analysis of the DLFM-CMDFC manner on the test CIFAR-10 dataset. The outcomes recognized that the DLFM-CMDFC approach has resulted in a proficient outcome with the decreased training and validation loss. It can be stated that the DLFM-CMDFC technique has obtainable minimum validation loss over the training loss.

The prec_*n*_ analysis of the DLFM-CMDFC technique with existing ones on the test dataset is given in Table 3.

Figure 12 illustrates the prec_*n*_ analysis of the DLFM-CMDFC technique with existing ones. The figure has shown that the IFD-AOS-FPM and CMFD-BMIF techniques have obtained reduced prec_*n*_ of 53.90% and 54.40%. At the same time, the CMFD and BB-KB-ICMFD techniques have resulted in moderate prec_*n*_ of 57.34% and 56.62%, respectively. Moreover, the CMFD-GAN-CNN technique has accomplished near optimal prec_*n*_ of 69.64%. However, the DLFM-CMDFC technique has resulted in superior performance with the prec_*n*_ of 97.27%.

Figure 13 illustrates the rec_*ll*_ analysis of the DLFM-CMDFC approach with current ones. The figure exhibited that the CMFD and CMFD-BMIF algorithms have obtained reduced rec_*ll*_ of 49.39% and 80.20%, respectively. Concurrently, the CMFD-GAN-CNN and BB-KB-ICMFD techniques have resulted in a moderate rec_*ll*_ of 80.42% and 80.40%, respectively. In addition, the IFD-AOS-FPM system has accomplished near optimal rec_*ll*_ of 83.27%. But, the DLFM-CMDFC technique has resulted in a maximal performance with the rec_*ll*_ of 96.46%.

Figure 14 depicts the *F*_score_ analysis of the DLFM-CMDFC system with present ones. The figure portrayed that the IFD-AOS-FPM and CMFD techniques have obtained reduced *F*_score_ of 54.39% and 49.26, respectively. Simultaneously, the CMFD-BMIF and BB-KB-ICMFD techniques have resulted in a moderate *F*_score_ of 59.43% and 60.55%, respectively. Also, the CMFD-GAN-CNN algorithm has accomplished near optimal *F*_score_ of 88.35%. Eventually, the DLFM-CMDFC manner has resulted in increased efficiency with the *F*_score_ of 96.06%.

The article "Design of Automated Deep Learning-Based Fusion Model for Copy-Move Image Forgery Detection" was retracted in 2023. Reasons: signs of a paper mill; suspected computer-generated content; unreliable results or conclusions; concerns about the data.

## 5. Conclusion

This article has presented an automated copy-move forgery detection and localization model, named DLFM-CMDFC. The proposed DLFM-CMDFC technique encompasses the fusion of GAN and DenseNet models. In DLFM-CMDFC technique, the two outcomes are combined into a layer to define the input vectors with the initial layer of the ELM classifier. Moreover, the optimal parameter tuning of the ELM technique takes place by the use of AFSA. The outcomes of the networks are fed as input to the merger unit. Lastly, the difference between the input and targets areas is identified in a forged image. The performance validation of the proposed manner takes place using two benchmark datasets. The proposed research work outperforms with 97.27% of precision, 96.46% of recall, and 96.06% of F-score. The experimental outcomes pointed out the supremacy of the proposed technique on the recently developed approaches. As a part of future scope, the detection performance can be improved by the use of generative adversarial network (GAN) model.

## Figures and Tables

**Figure 1:** Framework of GAN.

**Figure 2:** Flowchart of AFSA.

**Figure 3:** Sample image forgery detection results. (a) Original image. (b) Tampered image. (c) Localization image.

**Figure 4:** Result analysis of DLFM-CMDFC model on MNIST dataset.

**Figure 5:** ROC analysis of the DLFM-CMDFC model on the MNIST dataset.

**Figure 6:** Accuracy analysis of the DLFM-CMDFC model on the MNIST dataset.

**Figure 7:** Loss analysis of the DLFM-CMDFC model on the MNIST dataset.

**Figure 8:** Result analysis of the CIFAR-10 model on the DLFM-CMDFC dataset.

**Figure 9:** ROC analysis of the DLFM-CMDFC model on the CIFAR-10 dataset.

**Figure 10:** Accuracy analysis of the DLFM-CMDFC model on the CIFAR-10 dataset.

**Figure 11:** Accuracy analysis of THE DLFM-CMDFC model on THE CIFAR-10 dataset.

**Figure 12:** Precision analysis of DLFM-CMDFC technique with existing manners.

**Figure 13:** Recall analysis of DLFM-CMDFC technique with existing manners.

**Figure 14:** F-Score analysis of DLFM-CMDFC model with existing manners.

**Table 1:** Result analysis of DLFM-CMDFC model on MNIST dataset.

No. of runs	Precision	Recall	Accuracy	F-score
Run-1	96.38	93.71	94.29	95.98
Run-2	93.83	95.51	94.61	93.93
Run-3	93.54	97.30	94.88	97.19
Run-4	96.54	95.52	96.45	97.32
Run-5	96.80	97.43	96.87	94.69
**Average**	**95.42**	**95.89**	**95.42**	**95.82**

**Table 2:** Result analysis of the DLFM-CMDFC model on the CIFAR-10.

No. of runs	Precision	Recall	Accuracy	F-score
Run-1	96.52	96.15	96.36	96.66
Run-2	95.75	97.45	96.90	94.77
Run-3	97.98	96.68	97.00	96.57
Run-4	97.51	95.93	97.02	93.50
Run-5	97.46	96.50	97.35	94.52
Run-6	97.78	96.70	97.20	97.23
Run-7	97.71	96.03	97.22	96.86
Run-8	96.98	96.68	96.00	96.82
Run-9	97.31	95.73	96.82	96.51
Run-10	97.66	96.70	97.55	97.17
**Average**	**97.27**	**96.46**	**96.94**	**96.06**

The article "Design of Automated Deep Learning-Based Fusion Model for Copy-Move Image Forgery Detection" was retracted in 2023. Reasons: signs of a paper mill; suspected computer-generated content; unreliable results or conclusions; concerns about the data.

**Table 3:** Comparative analysis of DLFM-CMDFC mode with existing techniques.

Methods	Precision	Recall	F-score
CMFD	57.34	49.39	49.26
IFD-AOS-FPM	53.90	83.27	54.39
CMFD-BMIF	54.40	80.20	59.43
BB-KB-ICMFD	56.62	80.40	60.55
CMFD-GAN-CNN	69.63	80.42	88.35
DLFM-CMDFC	97.27	96.46	96.06

## Data Availability

The data used to support the findings of this study are available from the corresponding author upon request.
